# Pruning Growing Self-Organizing Map Network for Human Physical Activity Identification

**DOI:** 10.1155/2022/9972406

**Published:** 2022-01-03

**Authors:** Lingfei Mo, Hongjie Yu, Wenqi Hua

**Affiliations:** School of Instrument Science and Technology, Southeast University, Nanjing 210096, China

## Abstract

Human physical activity identification based on wearable sensors is of great significance to human health analysis. A large number of machine learning models have been applied to human physical activity identification and achieved remarkable results. However, most human physical activity identification models can only be trained based on labeled data, and it is difficult to obtain enough labeled data, which leads to weak generalization ability of the model. A Pruning Growing SOM model is proposed in this paper to address the limitations of small-scale labeled dataset, which is unsupervised in the training stage, and then only a small amount of labeled data is used for labeling neurons to reduce dependency on labeled data. In training stage, the inactive neurons in network can be deleted by pruning mechanism, which makes the model more consistent with the data distribution and improves the identification accuracy even on unbalanced dataset, especially for the action categories with poor identification effect. In addition, the pruning mechanism can also speed up the inference of the model by controlling its scale.

## 1. Introduction

Appropriate amount of exercise can promote human blood circulation, help bone and muscle growth, enhance cardiopulmonary function, and also prevent diabetes, hypertension, and other diseases [1, 2]. Therefore, human activity monitoring is necessary for human health management. However, if the assessment of the amount of exercise only depends on the personal impression, the evaluation results are inevitably too subjective. Therefore, a reliable human physical activity identification system is needed to identify the daily human movements. The development of microelectromechanical sensors, Internet of Things technology, and high-speed low-power communication networks makes it easier to implement the task of human physical activity identification by using wearable sensors to form a human sensor network. The wearable device can perform the all-weather and uninterrupted collection of the activity information of the wearing part without affecting the daily activities of the human body. A human sensor network composed of multiple wearable devices can estimate the pose of different parts of the human body as well as the heart rate or the respiratory rate of the human body [3], and the data collected by these devices can be transmitted to the cloud storage via the network for data analysis [4]. All-weather data collection means that a large amount of human activity data is produced by wearing sensors, which makes it possible to analyze human daily activity and evaluate human health.

In early research, only one sensor is used to identify human physical activity [5–7]. Then, a multisensor system is introduced into this area [8–10]. Also, deep learning [11–13] and ensemble learning [14, 15] have been introduced into this area. However, these research methods based on vision are easily restricted by many factors, such as object occlusion and light conditions, and are not conducive to the protection of users' privacy. What is more, Graph CNN [16–21] has been widely studied in this field, but GNN is generally for image data, video data, or skeleton data, which has the ability of representation learning, but large computational power and training data is necessary. Compared with these methods, sensors with high computing power, small size, and low cost make it possible for people to interact with these devices as a part of their daily life.

The identification task inevitably needs labels to determine the identification results, but unsupervised learning models without labeled data can be used during model training, which will greatly reduce the proportion of demand for labeled data in the process of training and using models. Therefore, unsupervised learning has been introduced to both feature extraction [22] and activity identification [23–27]. Multiple unsupervised learning algorithms such as *k*-means, Gaussian mixture model (GMM), hierarchical clustering, and density-based spatial clustering of applications with noise (DBSCAN) have been applied to human physical activity identification. But *k*-means, GMM, and hierarchical clustering all need to have prior knowledge about the number of the classes of the dataset, GMM can only perform well on dataset with Gaussian distribution, DBSCAN is not suitable to dataset with high dimension or uneven density. Besides, it is difficult to identify with a unified model because different people have different physical activity patterns. However, most of the existing models are offline training, so they cannot make adaptive adjustment to the new input data to realize online learning or incremental learning. This defect makes these models cannot perform well on different individuals. The Self-Organizing Map (SOM) network is an unsupervised learning algorithm proposed by the Finnish mathematician Kohonen in 1990 [28]. It is based on Hebb's learning rules and only updates the connection weights between neurons based on activated neurons. Since the algorithm was proposed, there have been various improvements made by scholars. The improvements are aimed at the network structure [29–31] and the learning mechanism [32–35]. The improvement of parameter initialization is also a research target [36, 37]. These rich SOM network variants show that the SOM network is exceedingly scalable. Compared with other classic unsupervised learning algorithms, SOM only needs little prior knowledge about the dataset, and it can deal with high-dimensional data well. The proposed model can perform well in the field of human physical activity identification when the data distribution is complex; the Growing SOM network (GSOM) can achieve the adaptive adjustment of network structure to obtain the most suitable network structure for specific dataset and make the topology of neural network more consistent with the distribution of dataset. Growing SOM has been widely used in the Internet of Things area, including sensor network communication [38], big data analysis [39], and data mining [40]. Growing SOM and its variants had been utilized widely because of their characteristics [41, 42]. It is suitable for tasks when the researchers have no idea about the data distribution [43, 44]. In addition, the characteristics of Growing SOM enable it to generate new network neurons for new samples to identify them and realize incremental learning without losing the original information.

In this paper, a Pruning Growing SOM (PGSOM) model is proposed based on GSOM. After an additional pruning mechanism is introduced, the redundant neurons will be deleted to reduce inference time and the storage space of the model under the premise of ensuring identification accuracy. The introduction of PGSOM not only reduce the dependence of human physical activity identification on labeled data and the prior knowledge of the exact number of the categories, but also adjust the structure of the model to fit the dataset better. Because the training cost of the model is not high and there are few super parameters, a robust model can be trained offline through grid search.

The organization of this article is as follows: firstly, the importance of this research and the related work of this area will be introduced; then the method used in this article will be explained in detail; after that, there is a simulation experiment and a real-world experiment that helps to show the characteristics of the method, and the results will be analysed; at last, a conclusion is proposed about this article.

## 2. Materials and Methods

### 2.1. PA Identification Diagram

The human physical activity identification is shown in Figure 1. In the experiment, the wearable device is used to obtain the activity data of different individuals. The input dataset is ready after feature extraction and feature selection, but different individuals' activity patterns are not consistent, and it is expensive to obtain a large quantity of labeled data in reality. What is more, it is difficult to design appropriate topology for different datasets. PGSOM could learn without supervision and be adjusted adaptively according to the scale and dimension of the dataset to reduce the quantization error. Then, a small amount of labeled data is used to calibrate the neurons in the trained network to obtain a model for the activity identification of different individuals.

### 2.2. SOM Network

The SOM network structure is shown in Figure 2. It is a feedforward neural network composed of an input layer and an output layer. The number of neurons in the input layer is the same as the dimension of the input sample. The output layer is also called the competition layer. Most of the neurons in the layer are arranged in two dimensions. The input layer and the output layer are fully connected networks with variable weights. The samples are input to the network for training, the neuron with the smallest Euclidean Distance from the input sample is the winner, and the weights of the neurons in the neighborhood of the winner are updated. The labeled information is not needed in training. After unsupervised training, a small number of labeled samples can be input to label the activated neurons.

The calibration algorithm is summarized as follows:

### 2.3. Growing SOM Network

The disadvantage of SOM is that it requires a preset network topology, and a large number of experiments are needed to find an appropriate network topology to the dataset.

The structure of GSOM starts with four neurons and grows on boundary based on heuristics and input representation. GSOM controls the difficulty of network growth by adjusting hyperparameters. When the cumulative quantization error (CEQ) on an activated neuron reaches the growth threshold (GT) and the winner neuron is a boundary neuron, it will perform growth operations; GT is a hyperparameter to control the ability about growth. Its CEQ will be halved and distributed to all adjacent neurons if it is not at the boundary of the network, which is shown in Figure 3.

However, GSOM also faces growth controllability issues. The increasing number of new neurons will contribute to the old neurons less activated because their weight vectors do not correspond to a certain pattern. Therefore, a pruning mechanism needs be introduced to optimize GSOM.

### 2.4. Pruning Growing SOM Network

Cutting the connection between neurons belonging to different patterns has been proved to be a way to adjust the network structure [45–47]. The key is to find a proper method to decide when a neuron (or the connection between neurons) should be removed.

The Pruning Growing Self-Organizing Map cuts neurons when the samples can activate the neuron being less than a predesigned threshold. When the dataset is unbalanced, samples of one or more categories are significantly less or more than others, the threshold is hard to be designed to make the pruning mechanism able to equally treat neurons represent minority category and majority category.

The TurSOM [48] uses neuron age threshold as the pruning threshold, but due to its mechanism, it prefers to cut new neurons, not the old neurons. This mechanism will make the newly input knowledge harder to be learned.

Inspired by the SOINN proposed by Furao and Hasegawa [49], a pruning mechanism based on the active degree of the neurons was proposed to improve GSOM. The inactive neurons in the GSOM contain very little useful information and have limited contribution to the performance of network by the theory of SOINN. The number of neurons can be effectively controlled without significantly affecting the accuracy of the model if the mechanism is added.

The algorithm uses neuron's age to describe how much time has passed since the neuron was last activated and it will eliminate neurons that have been inactive for a long time and preserve newborn neurons and the neurons that are often activated, which makes the model more suitable for learning new information without forgetting the useful information of the past; the pruning operation of PGSOM is shown in Figure 4. After the weight update and growth of the network are completed, all inactive neurons will be deleted.

Once an input sample *x* is presented to PGSOM, the index of the winner neuron is calculated according to (1) and (2) [28]. Then, the CEQ [29–31] is calculated by (3) and (4). Update the weights of the winner neuron and other neurons in its topological neighborhood according to (4) and (5).

(1) $$\begin{array}{c} d_{i}=x\left(t\right)-w_{i}{}^{2},\;\;i\in \phi \left(t\right), \end{array}$$

(2) $$\begin{array}{c} \text{winner}\left(t\right)=\arg\min\left\{d_{i}\right\}, \end{array}$$

(3) $$\begin{array}{c} {\text{CEQ}}_{\text{winner}\left(t\right)}={\text{CEQ}}_{\text{winner}\left(t\right)}+\;\eta \left(t\right)\times d_{i}, \end{array}$$

(4) $$\begin{array}{c} \eta \left(t+1\right)=\left(1-\left(\frac{R}{\left|\phi \left(t\right)\right|}\right)\right)\times \eta \left(t\right), \end{array}$$

(5) $$\begin{array}{c} w_{i}\left(t+1\right)=w_{i}\left(t\right)+\eta \left(t\right)\times \left(w_{\text{winner}\left(t\right)}\left(t\right)-w_{i}\left(t\right)\right)\times e^{-d_{i}},\;i\in \phi \left(t\right). \end{array}$$

The symbol *w* is the weight vector of neuron in competition layer; *d* is Euclidean distance between the weight vector of input sample and the weight vector of competition layer. Φ (*t*) is a set of all neurons in competition layer. *η* is decay factor, which decreases with the increase of iteration, and is used to ensure the training of PGSOM convergence. The network enters the growth stage after updating the weights.

Judging whether the CEQ of the winner neuron exceeds the growth threshold, the growth threshold can be determined by (6), *D* is the dimension of input sample, and spread factor (SF) is a hyperparameter between 0 and 1 to influence the difficulty of network growth. If the above condition is true and the winner is at the boundary of the network, the new neuron will be used to fill the surrounding of the winner neuron as (7) and (8) [29–31], and the weight of the new neuron is initialized by interpolation. If the winner neuron is not a boundary neuron, the CEQ is halved and the lost error is equally distributed to the neurons around as shown in Figure 3. Finally, the age of new neurons and winner neurons is updated to 0, and ages of the remaining neurons are increased by 1 as (9). At the same time, the neurons whose age exceeded the age threshold are deleted, which can be expressed by (10) and (11).

(6) $$\begin{array}{c} \text{GT}=-D\times \text{ln}\left(\text{SF}\right), \end{array}$$

(7) $$\begin{array}{c} \text{New neuron}\left(t\right)=\left\{\begin{array}{c} \text{neurons in remaining neighborhood,}\\ \text{if winner}\prime \text{s CEQ}\geq \text{GT and winner is at the boundary,}\\ \left\{\;\right\},\text{ else,} \end{array}\right) \end{array}$$

(8) $$\begin{array}{c} \phi \left(t\right)=\;\phi \left(t\right)\;\cup^{}\text{New neuron}\left(t\right), \end{array}$$

(9) $$\begin{array}{c} {\text{Age}}_{i}=\left\{\begin{array}{cc} 0, & \text{winner or new neuron,}\\ {\text{Age}}_{i}+1, & \text{else}, \end{array}\right) \end{array}$$

(10) $$\begin{array}{c} \text{Delete}\left(\text{t}\right)=\left\{neu_{i}|i\in \phi \left(t\right)\cap^{}\;{\text{Age}}_{i}>M\;\right\}, \end{array}$$

(11) $$\begin{array}{c} \phi \left(t+1\right)=\;\phi \left(t\right)-\text{Delete}\left(t\right). \end{array}$$

The training algorithm is summarized as follows:

## 3. Results and Discussion

### 3.1. Dataset Description

A total of 110 volunteers were called for data collection; each volunteer carried 5 to 7 physical activities [50]. The whole statistic characteristics of volunteers are given in Table 1.

The experiment involved a total of 9 common human activities; the label, kind, and the number of activities after feature engineering are shown in Table 2. All physical activity data come from two triaxial acceleration sensors worn on the wrist and hip and a piezo sensor worn on the abdomen, whose sampling frequency is 30 Hz; as shown in Figure 5, multiple raw data are stored in SD card for training model in offline environment. The raw data collected is shown in Figure 6.

A sliding window with length of 500 sampling points [51] is used to divide the raw data into several units. Each unit contains 7 signals combined with 6 signals from 2 triaxial acceleration sensors and one signal from a ventilation sensor; on this basis, we add 2 synthetic acceleration signals. The calculation formula of synthetic acceleration signal is as follows:

(12) $$\begin{array}{c} \text{synthetic signal}=\sqrt[{2}]{x^{2}+y^{2}+z^{2}}. \end{array}$$

11 features are extracted from each signal, respectively, as shown in Table 3, and the correlation coefficients between the synthetic acceleration signal from hip and piezo signal, the synthetic acceleration signal from wrist and piezo signal are calculated, which forms a 101-dimensional (11 *∗* 9 + 2 = 101) dataset.

## 4. Experiment and Results

One of the most important parameters of model is Age threshold (*M*), which determines the life cycle of neurons that have not been activated for a long time. The old neurons are more likely to be preserved with *M* increasing. Another important parameter is SF, which determines the growth threshold (GT) and affects the speed of the growing. 8586 samples are divided into training set and validation set in a ratio of 9 : 1; then, 10-fold cross validation is conducted. In each iteration of training, 4000 samples are randomly selected from 7727 samples for training, and fixed 2000 samples which are selected from current training set for calibration. The 859 samples in the validation set are used to evaluate the performance after each iteration of training. Ratio factor (RF) is the ratio of *M* to the size of samples in each iteration (batch size); for example, when the size of input in each iteration is 4000 and RF is 1.25, the *M* of neuron is 5000, as (13). First, the ratio factor is set as 1 and different SF used to verify the impact of SF on network size; the result is shown in Figure 7.

(13) $$\begin{array}{c} \text{RF}=\text{M}÷\text{ batch size.} \end{array}$$

When the growth and pruning of the network reach a balance, the network will converge. Therefore, comparative experiment is carried out on the basis of adjusting the two parameters, recording the accuracy of the PGSOM on the validation set and the number of neurons. The experimental results are shown in Figure 8. The training curve of the model that has high accuracy is shown in Figure 9.

As can be seen from Figure 8, the PGSOM achieves the highest accuracy when SF = 0.8 and RF = 1.5. It can be seen from the training curve in Figure 8 that PGSOM and GSOM models have begun to converge after 45 iterations, and PGSOM can achieve higher accuracy in the validation set. In order to verify the superiority of PGSOM, we compare PGSOM with SOM and GSOM. Experiments will be conducted on a personal computer with Intel® Core™ i5-10210U CPU, which is quad core, and the frequency is 1.60 GHz. The program used to train the models runs in the Python environment (Python 3.7). Indicators such as the accuracy of model, inference time, and the size of the model are used for comparing the performance of SOM series models. The comparison results are shown in Table 4. The hardware configuration of inference stage is consistent with that of training stage.

In addition, we supplement the comparison results between PGSOM and other unsupervised learning methods such as *k*-means, GMM, DBSCAN, and hierarchical clustering in Figure 10.

Other indicators such as kappa, recall, and *F* measure are calculated in Table 5.

## 5. Discussion

There will be isolated neuronal clusters no matter how to set the hyperparameter of PGSOM from Figure 7, which shows that there are transition regions between neurons representing different patterns, and the neurons in these transition regions are deleted because they cannot represent any pattern, pruning out the fact that these useless neurons will help speed up the training of the PGSOM, and the size of the PGSOM will increase with the increase of SF from (a) to (d) in Figure 7.

Then, different SF and RF are set up to train PGSOM to find the appropriate hyperparameter for the physical activity dataset and the best accuracy appears when SF = 0.8 and RF = 1.5 from Figure 8. In Figure 9, we draw several training curves of PGSOM and GSOM, which proves that the classification performance of PGSOM is better than GSOM, and each model basically converges when the number of iterations reaches 45. Therefore, in the following experiments, we set the maximum iterations as 50 to ensure the network convergence.

In Table 3, we compare the performance of a series of SOM networks including SOM of 3 structures (20 *∗* 20, 25 *∗* 25, and 30 *∗* 30), GSOM of 3 structures (SF = 0.75, 0.8, and 0.85), and PGSOM of 6 structures (SF, RF = 0.75/1.25, 0.75/1.50, 0.80/1.25, 0.80/1.50, 0.85/1.25, and 0.85/1.50) according to the accuracy of model, inference time, and the size of the model. Generally speaking, networks with more neurons have better identification ability and generalization performance, but it will also increase the cost of training and retain too many redundant neurons to increase the cost of model storage. The top accuracy of SOM is 86.723% when the size of competition layer is 30 *∗* 30, the top accuracy of GSOM is 88.272% when SF is 0.8 and the top accuracy of PGSOM is 90.120% when SF is 0.8 and RF is 1.5. Obviously, the last two models have better performance. The inference time of top PGSOM model is 0.262 ms, which is 50.3% less than the top GSOM model, and the number of neurons used is 856.1, which is 31.7% less than the top GSOM model. It proves that the introduction of pruning mechanism can effectively delete redundant neurons, improve the structure of the network, and optimize the training speed of the network.

Besides, both GSOM and PGSOM have the ability to grow new neurons when there are samples belonging to new patterns being input. The network will distribute new area to store these new patterns, which means these models have incremental learning ability. In Figure 10, it can be found from the experimental results that *k*-means algorithm performs worst among all unsupervised learning algorithms because it misidentifies Housekeeping and Playing tennis more frequently than other algorithms. All 6 algorithms have difficulty in distinguishing Walking and Running (low speed). Due to the length of the article, the confusion matrix of each algorithm is not expanded here. But since the activity category number is fixed, *k*-means, GMM, and hierarchical clustering algorithm cannot generate more clusters to describe these two activities more accurately. As for DBSCAN, the data density is obviously uneven in this dataset, especially those of easy-misidentified activity. Therefore, the performance of DBSCAN is limited. But GSOM and PGSOM can get over these adverse conditions to reach higher accuracy. In addition, because the adaptive adjustment mechanism of the network increases the stability of the network, the standard deviation of PGSOM is smaller than other unsupervised learning methods.

We give the confusion matrix of GSOM and PGSOM in Figure 11 to analyze the source of identification error and find that the main error source of both GSOM and PGSOM is the misclassification of Playing tennis as Playing basketball or Moving objects. We hold the view that it is due to the imbalance of the dataset, but the identification accuracy of other activities by PGSOM has reached a high level, which also reflects the robustness of the algorithm to the unbalanced dataset. And the identification effect of PGSOM is almost better than GSOM. We believe that the pruning mechanism removes redundant neurons and reduces the misidentification rate of the model.

The results of the experiments indicate that the proposed model works well in the human physical activity identification task, and the identification effect of action 2 and action 8 is significantly improved because of the pruning mechanism deleting a large number of ineffective neurons with side effects on identification. In addition, due to the incremental learning ability of PGSOM, this model can adapt itself to the particular user when practically applied, which means that individual differences will not be a serious problem when this model is utilized as a human physical activity classifier if each user uses its own physical activity data to further train this model.

## 6. Conclusions

PGSOM is proposed to address the scale of GSOM neurons. The adaptive growth of GSOM can adjust the structure of model to the distribution of the dataset with the limitations of little prior knowledge, which makes the application scenarios of the algorithm more abundant and makes it possible for the algorithm to migrate between different individuals. But it also leads to a large number of neurons, which increase the storage and reduce the inference speed and the identification accuracy of the model. PGSOM inherits the advantages of GSOM and adds pruning mechanism, which can delete the inactive neurons with useless information as well as learn the new knowledge. The PGSOM algorithm has been utilized to identify 9 kinds of physical activities and the accuracy on the provided dataset can reach 90.120%. Compared with other unsupervised learning algorithms, the proposed algorithm has competitive effect. Besides, it can obtain higher identification accuracy and reduce the inference time as well as reduce the storage cost of the model.

## Figures and Tables

**Figure 1:** Human physical activity identification with PGSOM.

**Figure 2:** SOM network structure. Different colours of neurons represent different clusters; each input sample can activate a neuron in output layer.

**Figure 3:** GSOM network structure and related operations. (a) New neurons grow at the dotted line position. (b) The cumulative error of winner neurons is halved and propagated to neurons; red neuron is the winner.

**Figure 4:** Pruning operation of PGSOM; the yellow neurons are older than age threshold.

**Figure 5:** Wearing position of sensors and raw data acquisition. The wrist unit and the abdominal unit transmit the sensor data to the hip unit wirelessly via ZigBee [50].

**Figure 6:** Sensor raw data. (a) Walking. (b) Running (low speed).

**Figure 7:** Neuron distribution of PGSOM with different spread factors. (a) SF = 0.1. (b) SF = 0.25. (c) SF = 0.5. (d) SF = 0.75.

**Figure 8:** Results under different SF and RF. (a) Accuracy of model. (b) Number of neurons in the model.

**Figure 9:** Training curve of Some models. (a) Accuracy of PGSOM. (b) Accuracy of GSOM.

**Figure 10:** Accuracy of unsupervised learning algorithms in proposed human physical activity dataset.

**Figure 11:** Confusion matrix of model. (a) Confusion matrix of top GSOM model. (b) Confusion matrix of top PGSOM model.

**Algorithm 1:** Class Calibration Algorithm.

**Algorithm 2:** Pruning Growing Self-Organizing Map.

**Table 1:** Volunteers' information.

Distribution			Time duration of each activity
Information	Category	Number		Percentage
Gender	F	59	53.6%	Each volunteer performs 5–7 kinds of physical activities for 5 minutes and rest for 2 minutes after each exercise to lower heart rate
	M	51	46.4%	
Age (years)	20–30	30	27.3%	
	30–40	28	25.5%	
	40–50	25	22.7%	
	50–60	27	24.5%	
Mass (kg)	<50	2	1.8%	
	50–60	26	23.7%	
	60–70	34	30.9%	
	70–80	13	11.8%	
	80–90	21	19.1%	
	>90	14	12.7%	
Height (cm)	150–160	16	14.5%	
	160–170	43	39.1%	
	170–180	33	30.0%	
	>180	18	16.4%	
BMI (kg/m^2^)	<18.5	1	0.9%	
	18.5–25	65	59.1%	
	25–30	30	27.3%	
	>30	14	12.7%	

**Table 2:** Physical activity and Label, and the number of each kind of samples after feature engineering.

	Label and activity	
1-Table working (1635)	2-Housekeeping (807)	3-Moving objects (794)
4-Walking (840)	5-Cycling (1549)	6-Running low speed (1646)
7-Running fast speed (494)	8-Playing tennis (359)	9-Playing basketball (462)

**Table 3:** All the extracted features.

Data sources	Features	Total number
Uniaxial signal and synthetic acceleration signal	Mean, variance, root mean square, kurtosis, skewness, energy [10, 25, 50, 75, and 90] percentile	11 *∗* 9
Between each synthetic acceleration signals and piezo signal	Correlation coefficient	2

**Table 4:** Training performance of different SOM models

Model	Hyperparameter	Accuracy (%)	Inference time (ms)	Number of neurons
SOM	20 *∗* 20	79.269	0.071	400
	25 *∗* 25	84.405	0.110	625
	30 *∗* 30	**87.596**	0.261	900
GSOM	SF = 0.75	87.713	0.294	1044
	SF = 0.80	88.027	0.315	1155
	SF = 0.85	**88.272**	0.527	1254
**PGSOM (ours)**	SF = 0.75, RF = 1.25	88.644	0.127	731
	SF = 0.75, RF = 1.50	88.994	0.161	797.1
	SF = 0.80, RF = 1.25	89.401	0.265	864
	SF = 0.80, RF = 1.50	**90.120**	0.262	856.1
	SF = 0.85, RF = 1.25	89.809	0.261	864
	SF = 0.85, RF = 1.50	89.762	0.283	929

**Table 5:** Performance comparison of unsupervised learning algorithms.

Algorithm	Kappa	*F* measure	Inference time (ms)
GSOM	0.882	0.896	0.527
**PGSOM (ours)**	0.897	0.902	0.262
*k*-means	0.611	0.613	4.101
GMM	0.852	0.873	9.033
Hierarchical cluster	0.802	0.786	4.371
DBSCAN	0.778	0.808	4.205

## Data Availability

The human activity data used to support the findings of this study are available from the corresponding author upon request.
